# Growth Differentiation Factor-15 Based ABC (Age, Biomarkers, Clinical History)-AF (Atrial Fibrillation)-Bleeding Risk Score for Elderly Patients with Nonvalvular Atrial Fibrillation

This article has been retracted.

**DOI:** 10.1155/2022/2863815

**Published:** 2022-03-08

**Authors:** U Fan O, Tou Kun Chong, Yulin Wei, Cheok Ian Lo, Wei Wu

**Affiliations:** ^1^Department of Cardiology, Sun Yat-sen Memorial Hospital of Sun Yat-sen University, Guangzhou, Guangdong Province, China; ^2^Department of Cardiology, Kiang Wu Hospital, Macau Special Administrative Region, Macao, China

## Abstract

**Background:**

Growth differentiation factor-15 (GDF-15) is a strong predictor of bleeding in atrial fibrillation (AF) patients. The novel ABC (age, biomarkers, and clinical history), AF, and bleeding risk score outperforms HAS-BLED bleeding risk score for major bleeding (MB) in patients with AF receiving oral anti-coagulation in the clinical trial cohort. However, it has not been entirely externally validated. We aimed to refine and understand the application of the ABC-AF bleeding risk score in elderly (aged ≥65 years old) patients with nonvalvular atrial fibrillation (NVAF) for predicting the different types of bleeding events and anti-thrombotic treatments.

**Methods:**

We identified elderly patients with NVAF between March 2018 and December 2019 who were hospitalized for the first time after a diagnosis of NVAF. We measured the plasma concentration of the ABC biomarkers (growth differentiation factor 15 (GDF-15) and cardiac troponin-T (cTnT)) from enrolled patients. We collected their general information and follow up for one year until December 2020. During the follow-up period, information on the occurrence of bleeding events (major bleeding, clinically relevant nonmajor gastrointestinal bleeding (CRNM GIB), and minor bleeding events) was collected.

**Results:**

We enrolled 342 elderly NAVF patients; the ABC-AF bleeding and HAS-BLED scores were quantified. With an average of 1.5 years of follow-up, 6 patients had an intracranial hemorrhage; 57 patients had CRNM GIB; and 68 patients had minor bleeding events (36 fecal occult blood positive and 32 other minor bleeding events). The ABC-AF bleeding score yielded a C-index of 0.72 (95% CI 0.60–0.84) for predicting MB in elderly patients with NAVF, C-index of 0.69 (95% CI 0.57–0.82) by HAS-BLED score. Comparison of the incidence of bleeding events during follow-up and the predicted 1-year incidence of bleeding events by each bleeding risk score, ABC-AF bleeding, and HAS-BLED scores have similar value in predicting the risk for elderly patients with NAVF in different types of bleeding events, whether on oral anti-coagulation treatment (OAC) or non-OAC (*P* > 0.05).

**Conclusion:**

In elderly patients with NVAF, the biomarker-based ABC-AF bleeding score showed similar performance compared with the HAS-BLED bleeding risk score.

## 1. Introduction

The benefit of oral anti-coagulation in patients with nonvalvular atrial fibrillation (NVAF) is based on a balance between reduction in stroke and bleeding events. Bleeding risk increasing has become one of the concerns affecting the popularization of anti-coagulation therapy, especially in elderly patients. Bleeding/stroke risk scores stratification can guide appropriate anti-coagulation and balance the risk of bleeding/embolism. HAS-BLED bleeding risk score is one of the commonly used scores recommended by the guidelines for managing NVAF. However, HAS-BLED bleeding risk score based on clinical factors for predicting bleeding risk with a C-index of approximately 0.60–0.65 [1]. Due to the limited capacity of clinical risk scores, the use of biomarkers might be an attractive tool to improve clinical risk stratification.

Growth differentiation factor-15 (GDF-15) is a novel cardiac biomarker [2, 3], a strong predictor of bleeding in patients with NVAF, and evaluates bleeding, stroke, and death risk in atrial fibrillation (AF) [4–6]. Studies [6–8] showed that GDF-15 has better stability and continuity as a novel cardiac biomarker, which has become a hotspot of clinical research for bleeding risk evaluation and clinical application in patients with atrial fibrillation [9, 10]. The novel ABC (age, biomarkers, and clinical history) AF bleeding risk scores outperform the HAS-BLED bleeding risk score for major bleeding (MB) patients with NVAF receiving oral anti-coagulation in the clinical trial cohort such as ARISTOTLE [6], RE-LY [6], and ENGAGE AF-TIMI 48 [8] indicated that the ABC-AF bleeding risk score outperformed the traditional HAS-BLED score. The ABC-AF bleeding score was recommended in European atrial fibrillation management guidelines [7] since 2016.

However, it has not been entirely externally validated, such as comparing different bleeding risk scores under different anti-thrombotic strategies or evaluating the predictive ability of bleeding risk scores under various degrees of bleeding events. The objective of our study was to analyze the predictive performance of the ABC-AF bleeding compared to HAS-BLED score for major bleeding (MB) [11], clinically relevant nonmajor gastrointestinal bleeding (CRNM GIB) [12] events, and minor bleeding events in elderly NVAF patients.

The occurrence of bleeding events with anti-thrombotic therapy is often the result of multiple factors. A series of assessment methods have been developed to assess bleeding risk. However, since the population for which the score is established is mainly based on European and American populations and studies based on Asian populations are lacking, the efficacy of assessing bleeding risk in Chinese people needs further observation. At the same time, for the elderly who need anti-thrombotic therapy, the role of these scores needs to be further verified. We need to combine domestic research data to develop a group scoring system for these scores. With awareness of the differences in the responsiveness-benefit profile of East Asian and Western populations to anti-thrombotic drugs, a simple application of clinical data based on Western people to guide anti-thrombotic therapy in East Asian populations Thrombosis can be uncomfortable. New evaluation methods need to be verified and explored in future research.

## 2. Methods and Material

A prospective observational study was conducted between March 2018 and December 2019. Consecutive patients were collected from the Department of Cardiology, Kiang Wu Hospital, Macau Special Administrative Region (Macau SAR). We utilized an electronic healthcare information system (HIS) to gather all medical information of patients who received medical care in either in- or out-patient settings. All eligible patients are Macau native residents of Chinese nationality and aged ≥65 years, diagnosed with NVAF (ICD-10: I48.0–148.9) via either a 12-lead electrocardiogram (ECG) or 24-hour ECG monitor (Holter), and were included in the analysis. Of 368 screened patients, 26 were excluded, and 342 patients were eventually enrolled in this study (Figure 1). The Scientific Ethics Committee approved the study protocol of Kiang Wu Hospital of Macau (Approval no. 2017–001).

### 2.1. Blood Samples and Laboratory Analysis

We measured the plasma concentration of the ABC-AF biomarkers (N-terminal pro-B-type natriuretic peptide (NT-proBNP), cardiac troponin-T (cTnT), and GDF-15). Plasma concentrations of GDF-15, NT-proBNP, and cTnT were measured centrally with the Elecsys GDF-15 commercial assay kit (Roche Diagnostics) [13]. All patients selected for the study were drawn venous blood within 48 hours of admission. The test was performed on the Roche analyzer Cobas e601 (Roche Diagnostics) system. The plasma GDF-15 (detection range: 0–0,000 pg/mL), NT-proBNP (detection range: 5–35,000 pg/mL), and high sensitively cTnT (cTnT, hs-cTnT) (detection range: 0.03–10.0 ng/mL) were performed on the Roche analyzer Cobas e601 (Roche Diagnostics) system.

### 2.2. Study Population

All enrolled patients were elderly NVAF patients who survived more than one year after being registered. Patients were included with (1) age ≥65 years old with a diagnosis of NVAF, (2) Chinese native resident in Macau, and (3) agree to regular follow-up visits and blood tests. Patients with (1) valvular AF such as postmechanical valve replacement or moderate to severe rheumatic mitral valve stenosis; (2) AF caused by reversible factors including acute myocardial infarction, acute myocarditis, pericarditis, pulmonary embolism, electrocution, or binge drinking; (3) any primary coagulation disorders; (4) malignant tumor or blood disease; (5) died within one week of enrollment; (6) lost to follow-up within one year of follow-up; and (7) patients self-adjust anti-coagulation strategy during follow-up due to poor patient compliance were excluded.

### 2.3. Definition

- Elderly [14]: as a convention, a person aged 65 years or more is referred to as “elderly.”
- NOACs: Nonvitamin K antagonist oral anticoagulants (NOACs) are a class of drugs that directly inhibits the activity of specific “targeted” coagulation factors which inhibit thrombin (dabigatran) and factor Xa (rivaroxaban, apixaban, and edoxaban).
- OACs: Oral anticoagulants (OACs) using either vitamin K antagonists (VKAs, warfarin) or NOACs.
- Major bleeding (MB) [11]: Major bleeding was bleeding that was fatal or requiring transfusion of at least two units packed blood cells or overt bleeding with a drop in hemoglobin concentration of at least 20 g/L or hemorrhage into a critical anatomical site (e.g., intracranial, retroperitoneal).
- CRNM (clinically relevant nonmajor) GIB [12]: The International Society defined bleeding on thrombosis and hemostasis (ISTH) classification as any bleeding requiring medical intervention by a healthcare professional or leading to hospitalization or increased concentration of care, which did not fit the criteria for major bleeding. And CRNM GIB was defined as gastrointestinal bleeding (GIB) that meets the classification of CRNM bleeding.
- Minor bleeding [15]: Minor bleeding was defined as every overt bleeding that does not fulfill the criteria of MB or CRNM bleeding, according to the ISTH, for example, subconjunctival hemorrhage, dental bleeding, epistaxis, hemorrhoidal bleeding, extremity bruising, self-limited epistaxis, and also fecal occult blood (OB) positive. Most minor bleeding is OB positive in clinical practice, so it was analyzed independently in this study. Another minor bleeding represents minor bleeding except for OB positive.
- HAS-BLED score [16]: H, hypertension (uncontrolled systolic blood pressure >160 mmHg); A, abnormal renal or liver function; S, previous stroke; B, bleeding history; L, labile international normalized ratio (only applies to a vitamin K antagonists user); E, elderly (age ≥65 years), and D, concomitant drugs (anti-platelet or nonsteroidal anti-inflammatory drugs) or alcohol excess. HAS-BLED categories were defined as low/medium risk (0–2 points) and high risk (≥3).
- ABC-AF bleeding score [16]: Using GDF-15, cTnT, and hemoglobin (HB) as biomarkers and an Excel-based calculator according to the modified nomogram proposed by Hijazi et al., the ABC-AF bleeding risk categories were calculated according to the correlation between total points of nomograms with one-year risk of MB, which was defined as low/medium risk (0–2% predicted one-year risk of bleeding) and high risk (>2% indicated the one-year risk of bleeding).

### 2.4. Follow-Up and Clinical Bleeding Outcomes

We collected patients' demographic data and medical history, including hypertension, coronary artery disease, diabetes mellitus, heart failure, renal function, previous stroke/transient ischemic attack (TIA), peripheral arterial disease (PAD), and bleeding events, especially MB and CRNM GIB. We documented all the dosages and duration of anti-coagulant medication, comorbidities, laboratory data, ECG, and X-ray reports. Each patient in this research was tracked via the HIS until the patient developed bleeding or death events. In addition, all information related to anti-coagulant treatment and clinical bleeding, including MB, CRNM GIB, OB positive, and other minor bleeding events, were collected.

### 2.5. Statistical Analysis

Demographics and other baseline characteristics were described using frequencies for categorical variables and median and 24^th^ and 75^th^ percentiles for continuous variables. We used the Pearson chi-squared test to compare proportions. Receiver-operating characteristic curves (ROC) were performed for the ABC-AF bleeding and HAS-BLED scores to evaluate their predictive ability through C-index for survival data. *P-*value of <0.05 was defined as significant in statistical inference tests. The statistical analyses were performed with medicals and IBM SPSS statistics.

## 3. Results

### 3.1. Clinical Characteristics

A total of 342 elderly (≥65 years old, mean age 79.16 ± 8.72 years) patients with NVAF, 160 (46.78%) were male, and 109 (31.87%) were very elderly (≥85 years old). The median follow-up was 19.92 ± 6.83 (12.00–29.34) months. Baseline clinical and demographic characteristics are listed according to anti-coagulants treatment group as summarized in Table 1. All enrolled patients in the study have anti-coagulant therapy indications. Among them, 36 (11.11%) patients received no anti-thrombotic treatment (NAT); 134 (41.36%) patients received anti-platelet therapy (AP; aspirin 100 mg QD or clopidogrel 75 mg QD); 30 (9.26%) patients received VKA treatment; 142 (43.83%) patients received NOACs treatment of which 43 (13.27%) cases received dabigatran 110 mg BID, 40 (12.35%) cases rivaroxaban 15 mg QD, 46 (14.20%) cases apixaban 2.5 mg BID, and 13 (4.01%) cases edoxaban 30 mg QD. The average concentration of GDF15 is 4,610.85 ± 4,513.30 ng/L; ABC-AF bleeding risk score predicts a one-year risk of MB that was 5.16%. The detailed results are shown in Table 1.

### 3.2. Bleeding Outcomes

A total of 131 (38.30%) patients experienced any bleeding events. There were 6 (1.75%) patients who had experienced MB events (all of the 6 cases were suffered intracranial hemorrhage); 57 (16.67%) patients had CRNM GIB; 36 (10.53%) patients had fecal occult blood positive; and 32 (9.36%) patients had other minor bleeding events—grouped by anti-thrombotic strategy (NAT, AP, VKA, and NOACs), the occurrence of different bleeding events are grouped in Table 2. The results showed that the difference in MB, CRNM GIB, and OB positive among different anti-thrombotic strategies is not statistically significant. However, other minor bleeding events that occurred in the VKA group had seemed more (*P* < 0.05).

### 3.3. Comparison of ABC Bleeding Risk Score and HAS-BLED Bleeding Risk Score

The distribution of bleeding events according to the bleeding risk scores and GDF-15 concentration are shown in Table 3. During the follow-up, more than 80% of patients with MB, CRNM GIB, and OB positive were rated as high-risk group in either ABC-AF bleeding or HAS-BLED scores. Using Cox regression analyses, a HAS-BLED score ≥3 was associated with a 2.42-fold greater hazard for MB (HR 2.42, 95% CI 1.95–2.99, *P* < 0.001), whereas ABC-AF bleeding high-risk score category was associated with a 1.21-fold greater hazard for MB (HR 1.21, 95% CI 1.15–1.28, *P* < 0.001).

The GDF-15 concentration in the study enrolled elderly patients with NVAF was 4,610.85 ± 4,513.30 pg/mL. Among them, compared with the GDF-15 concentration in patients with any bleeding events (6,047.87 ± 5,346.50 pg/mL), those patients without bleeding events were lower GDF-15 concentration (3,718.67 ± 3,646.01 pg/mL, *P* < 0.05). The results also showed that there does not seem to be a significant correlation between the GDF-15 concentration and the severity of bleeding events (*r* = 0.230, *P* = 0.053).

Bleeding risk scores are used to predict the risk of bleeding after anti-coagulation therapy. Because the elderly patients included in this study are not all receiving anti-coagulation therapy, such as patients taking AP or NAT, such patients were classified as a non-OAC group; in contrast, patients with VKA or NOACs were classified as OAC group. Data presented according to the anti-thrombotic regimen (OAC and non-OAC) show the results in Table 4. Analysis of all enrolled elderly NVAF patients showed that the ABC-AF bleeding score yielded a C-index of 0.72 (95% CI 0.60–0.84) for predicting MB in elderly patients with NAVF, which yielded a C-index of 0.69 (95% CI 0.57–0.82) by HAS-BLED score (Figure 2). The Delong test compares the area under the ROC curve (AUC); the results suggest the difference between the ABC-AF bleeding scores, whether MB, CRNM GIB, OB positive, or even minor bleeding events; the traditional HAS-BLED score did not show statistical significance. Further analysis of the OAC and non-OAC subgroups, compared with two different bleeding risk scores in different subgroups, also indicated the AUC value difference between the ABC-AF bleeding score and the HAS-BLED score was not statistically significant. It evaluates the clinical usefulness of using the ABC-AF bleeding score for MB and CRNM GIB in real-world practice.

## 4. Discussion

GDF-15 [17] is a novel cardiac biomarker. As a nonspecific stress factor, GDF-15 is related to tissue damage and remodeling of inflammation, hypoxia, and cardiovascular disease [18]. Its plasma concentration significantly increases rapidly under the above-mentioned pathological conditions. Some studies [19, 20] show that GDF-15 concentrations are positively correlated with the severity of cardiovascular diseases (especially atrial fibrillation, non-ST segment elevation myocardial infarction, heart failure, etc.). In atrial fibrillation, GDF-15, NT-proBNP, and cTnT have been included in the European guidelines for managing atrial fibrillation, as an essential part of the ABC-AF bleeding risk score, providing clinical services beyond the HAS-BLED bleeding risk stratification. The effective supplement is used to guide the adjustment of anti-coagulant medication strategy. The purpose of this study is to conduct a preliminary discussion on the application of GDF-15 in the bleeding risk assessment of elderly patients with NVAF. In clinical practice, compared with HAS-BLED score, patients with ABC-AF bleeding score can be assessed more precisely and quantitatively, and “real” high-risk patients can be screened out of patients with the same risk stratification.

Similarly, because the ABC-AF bleeding risk score is dynamic linear and continuous, the evaluation of repeatable monitoring will bring new strategic guidance for assessing the risk change of the same patient after diagnosis and treatment. And it has been widely reported [21] that GDF-15 combined with TnT and NT-proBNP can further evaluate the prognosis of cardiology patients from the patient's overall state and will become the focus of future research. Cardiac-biomarker-based risk model will become a new way to predict risk and risk stratification of patients with NVAF in the future. Thus, the new ABC-AF bleeding risk score performed better than the HAS-BLED score in the ARISTOTLE [22] and RE-LY [23] clinical trials. A recent study [13] reported that the ABC-AF bleeding score yielded a C-index of 0.76 (95% CI, 0.71–0.81) in the aspirin cohort and 0.73 (95% CI, 0.69–0.77) in the combined anti-platelet cohort. The ABC-AF bleeding score outperformed the HAS-BLED score, which had a C-index of 0.61 (95% CI, 0.53–0.68) and 0.60 (95% CI, 0.55–0.65), respectively (*P* < 0.001 for both comparisons). However, the Murcia Atrial Fibrillation Project study reported that the HAS-BLED score gave an approximate net benefit of 4% over the ABC-AF bleeding score. Differences in risk scores between studies may be related to background factors [19] such as population, region, treatment strategy, anti-coagulation strategy, and patient age. At present, many clinicians are more interested in the real-world situation of the elderly receiving anti-coagulation therapy, which is the purpose of this study. Notably, this study indicated that the GDF-15 biomarker-based ABC-AF bleeding risk score and traditional bleeding risk scoring method correlate well for predictive bleeding risks of MB, CRNM GIB, and OB positive. Due to the small sample size in this study, the prediction of GDF-15 and the bleeding outcome of patients with atrial fibrillation still needs further investigation, including dynamic monitoring of the relationship between the evolution of GDF-15 in the course of disease diagnosis and treatment and the prognosis, and GDF-15 as a nonspecific biomarker, with the deepening of research. It is believed that GDF-15 can assist specific cardiac biomarkers such as NT-proBNP and cTnT in establishing a prediction model to guide clinical diagnosis and treatment strategies. GDF-15 also has a particular value for stroke risk prediction and prognostic risk score. With further research, it is expected that GDF-15 will develop more excellent clinical application value. Therefore, our findings in conjunction with the clinical information and stroke/prognosis score are the next step to personalized so-called precision medicine for balancing stroke/bleeding/prognosis in elderly patients with NVAF.

As a novel cardiovascular disease biomarker, GDF-15 has essential value in NVAF for risk stratification and prognostic evaluation. However, some issues still need further research and discussion, including determining the threshold in different diseases, balancing the sensitivity and specificity of the threshold, and how to use existing biomarkers to guide treatment strategies. At present, HAS-BLED, ORBIT, and other scores only provide references for high-risk bleeding factors, and the score level does not affect clinical decision-making. The ABC bleeding score, composed of biomarkers such as GDF-15, uses quantitative indicators to be more objective and quantitatively monitored. The dynamic data of the ABC bleeding score is easier to obtain, and with the development of big data, its predictive value will further increase. As a part of precision medicine in the future, it has excellent development potential.

In summary, the results in this study suggest that the GDF-15 concentration of elderly patients with NVAF is higher than the normal reference value (1200 pg/mL). Patients with bleeding events during follow-up had higher levels of GDF-15; it seems that GDF-15 concentration may have a predictive value for bleeding risks. The GDF-15 based ABC-AF bleeding risk score has equal ability to predict bleeding risk as to the HAS-BLED bleeding risk score.

The main limitations of this study are related to its retrospective nature and possible selection bias. To ensure the integrity of the risk factor assessment and other clinical data, we included only the patients from a southern Chinese population in the Macau Special Administrative Region (Macau SAR) of China. The results from our study warrant further validation by multicenter, prospective trials to further define the roles of OACs in a large scale of elderly patients with diversity in ethnicity, gender, and age.

## 5. Conclusion

In elderly NVAF patients, the GDF-15 based ABC-AF bleeding risk score has equal ability to predict bleeding and the HAS-BLED bleeding risk score.

## Figures and Tables

**Figure 1:** Flowchart of enrollment of the study. Of 368 subjects with atrial fibrillation who were aged ≥65 years old, we identified 342 eligible issues with nonvalvular atrial fibrillation. The ABC-AF and HAS-BLED bleeding scores were quantified. All enrolled subjects were followed for at least one year for various degrees of bleeding events (including major bleeding, clinically relevant nonmajor gastrointestinal bleeding, fecal occult blood positive, and other minor bleeding).

**Figure 2:** Receiver-operating characteristic curves (ROC) of HAS-BLED and ABC-AF bleeding scores for bleeding outcomes in all enrolled elderly NVAF patients. NVAF, nonvalvular atrial fibrillation; MB, major bleeding; CRNM GIB, clinically relevant nonmajor gastrointestinal bleeding; OB positive, fecal occult blood positive.

**Table 1:** Baseline characteristics.

Variable	All, *n* = 342	NAT, *n* = 36	AP, *n* = 134	VKA, *n* = 30	NOACs, *n* = 142
Age, years	79.16 ± 8.72	81.17 ± 10.76	79.06 ± 8.91	78.63 ± 7.69	78.87 ± 8.17
Group 65–74, *n* (%)	112 (32.75)	11 (30.56)	46 (34.33)	9 (30.00)	46 (32.39)
Group 65–74, years	68.97 ± 3.00	68.18 ± 3.57	68.72 ± 3.15	69.67 ± 3.04	69.28 ± 2.72
Group 75–84, *n* (%)	121 (35.38)	9 (25.00)	44 (32.84)	14 (46.67)	54 (38.03)
Group 75–84, years	79.45 ± 2.73	78.33 ± 2.78	79.91 ± 2.81	79.21 ± 2.91	79.31 ± 2.61
Group ≥85, *n* (%)	109 (31.87)	16 (44.44)	44 (32.84)	7 (23.33)	42 (29.58)
Group ≥85, years	89.32 ± 3.21	91.69 ± 3.30	89.02 ± 3.21	89.00 ± 2.89	88.79 ± 2.94
Male, sex, *n* (%)	160 (46.78)	8 (22.22)	69 (51.49)	9 (30.00)	74 (52.11)
Previous bleeding, *n* (%)	0 (0)	0 (0)	0 (0)	0 (0)	0 (0)
Previous stroke, *n* (%)	56 (16.37)	1 (2.78)	25 (18.66)	5 (16.67)	25 (17.61)
Previous TIA, *n* (%)	32 (9.36)	2 (5.56)	14 (10.45)	2 (6.67)	14 (9.86)
Heart failure, *n* (%)	162 (47.37)	9 (25.00)	57 (42.54)	24 (80.00)	72 (50.70)
Hypertension, *n* (%)	304 (88.89)	33 (91.67)	121 (90.30)	25 (83.33)	125 (88.03)
Diabetes, *n* (%)	131 (38.30)	7 (19.44)	62 (46.27)	12 (40.00)	50 (35.21)
Coronary artery disease, *n* (%)	148 (43.27)	6 (16.67)	81 (60.45)	8 (26.67)	53 (37.32)
Chronic kidney disease, *n* (%)	108 (31.58)	11 (30.56)	45 (33.58)	14 (46.67)	38 (26.76)
Peripheral arterial disease, *n* (%)	18 (5.26)	2 (5.56)	7 (5.22)	2 (6.67)	7 (4.93)
Hemoglobin (g/L)	115.65 ± 21.48	108.19 ± 23.55	114.65 ± 20.63	106.57 ± 22.32	120.39 ± 20.46
NT-proBNP (pg/mL)	4,925.88 ± 9,339.50	4,238.57 ± 9,798.98	5,698.02 ± 10,484.23	7,949.40 ± 11,013.76	3,731.99 ± 7,376.84
cTnT (ng/mL)	0.12 ± 0.55	0.31 ± 1.50	0.11 ± 0.32	0.13 ± 0.18	0.07 ± 0.23
GDF-15 (pg/mL)	4,610.85 ± 4,513.30	4,138.94 ± 4,221.84	5,302.78 ± 4,844.91	6,259.43 ± 6,490.14	3,729.25 ± 3,487.33
Group 65–74 (pg/mL)	3,674.68 ± 4,494.31	1,917.00 ± 1,901.88	4,554.96 ± 5,072.16	4,882.22 ± 6,092.32	2,971.15 ± 3,788.10
Group 75–84 (pg/mL)	4,506.32 ± 3,997.35	5,111.22 ± 4,640.24	4,838.43 ± 4,140.50	5,145.57 ± 4,125.49	3,969.17 ± 3,780.08
Group ≥85 (pg/mL)	5,691.91 ± 4,867.80	5,119.63 ± 4,741.36	6,548.95 ± 5,111.54	10,257.86 ± 9,634.98	4,251.07 ± 2,569.64
CREA (umol/L)	130.38 ± 126.40	126.67 ± 129.60	155.57 ± 172.78	160.10 ± 112.94	101.06 ± 43.97
ALT (u/l)	30.24 ± 86.95	25.17 ± 55.60	34.70 ± 80.22	22.33 ± 15.68	28.97 ± 106.69
CHA_2_DS_2_-VASc score	5 (4, 6)	4 (3, 5)	5 (4, 6)	5 (4, 7)	5 (4, 6)
HAS-BLED score	3 (2, 4)	2 (2, 4)	3 (3, 4)	3 (2, 4)	3 (2, 4)
ABC-stroke score with OAC (%)	1.53 (0.83, 3.07)	—	—	2.76 (1.71, 3.69)	1.43 (0.93, 2.53)
ABC-stroke score with non-OAC (%)	4.59 (2.49, 9.21)	2.54 (1.48, 5.45)	4.70 (2.24, 9.69)	—	—
ABC-AF bleeding score (%)	5.16 (2.71, 10.56)	4.78 (1.93, 14.24)	6.01 (2.69, 12.58)	7.99 (5.16, 12.70)	4.23 (2.68, 7.86)

Continuous variables are summarized as median (first quartile-third quartile). ABC indicates Age, Biomarkers, Clinical History; AF, atrial fibrillation; TIA, transient ischemic attack; NT-proBNP, N-terminal pro-B-type natriuretic peptide; cTnT, cardiac troponin *T*; GDF-15, growth differentiation factor; CREA, creatinine; ALT, alanine aminotransferase; NAT, no antithrombotic treatment; AP, antiplatelet; VKA, vitamin K antagonists; NOACs, non-vitamin K antagonist.

**Table 2:** Bleeding events in elderly NVAF patients with different antithrombotic strategies *n* (%).

Variable	All *n* = 342	NAT *n* = 36	AP *n* = 134	VKA *n* = 30	NOACs *n* = 142	2	*P*-value
Major bleeding	6 (1.75)	0 (0)	2 (1.49)	1 (3.33)	3 (2.11)	1.236	0.744
CRNM GIB	57 (16.67)	7 (19.44)	28 (20.90)	3 (10.00)	19 (13.38)	3.990	0.263
OB positive	36 (10.53)	4 (11.11)	14 (10.45)	4 (13.33)	14 (9.86)	0.332	0.954
Other minor bleeding	32 (9.36)	2 (5.56)	9 (6.72)	8 (26.67)^†§^	13 (9.15) ^△^	12.320	0.006

NVAF, nonvalvular atrial fibrillation; MB, major bleeding; CRNM GIB, clinically relevant nonmajor gastrointestinal bleeding; OB positive, fecal occult blood positive; NAT, no antithrombotic treatment; AP, antiplatelet; VKA, vitamin K antagonists; NOACs, non-vitamin K antagonist; † compared with NAT, *P*-value <0.05; § compared with AP, *P*-value <0.05; △ compared with VKA, *P*-value <0.05.

**Table 3:** Distribution of bleeding events according to the bleeding risk scores categories *n* (%).

		ABC-AF bleeding score		HAS-BLED score	
	N	GDF-15 (pg/mL)	Low/medium risk	High risk	Low/medium risk	High risk
Non-bleeding events	211 (100)	3,718.67 ± 3,646.01	47 (22.27)	164 (77.73)	87 (41.23)	124 (58.77)
All bleeding events	131 (100)	6,047.87 ± 5,346.50	12 (9.16)	119 (90.84)	26 (19.85)	105 (80.15)
Major bleeding	6 (100)	5,256.17 ± 3,857.65	0 (0)	6 (100)	0 (0)	6 (100)
CRNM GIB	57 (100)	7,396.96 ± 5,747.45	2 (3.51)	55 (96.49)	3 (11.54)	54 (94.74)
OB positive	36 (100)	6,159.11 ± 5,790.49	4 (11.11)	32 (88.89)	6 (23.08)	30 (83.33)
Other minor bleeding	32 (100)	3,668.09 ± 3,258.10	6 (18.75)	26 (81.25)	17 (65.38)	15 (46.88)

Note: NVAF, nonvalvular atrial fibrillation; MB, major bleeding; CRNM GIB, clinically relevant nonmajor gastrointestinal bleeding; OB positive, fecal occult blood positive; NAT, no antithrombotic treatment; AP, antiplatelet; VKA, vitamin K antagonists; and NOACs, non-vitamin K antagonist.

**Table 4:** Bleeding events and C-index of bleeding risk scores in elderly patients with NVAF, *n* (%).

Variable		ABC-AF bleeding score^#^	HAS-BLED score^#^	Z statistic	*P*-value
Overall (*n* = 342)	
Major bleeding	6 (1.75)	0.72 (0.60–0.84)	0.69 (0.57–0.82)	0.253	0.800
CRNM GIB	57 (16.67)	0.77 (0.70–0.84)	0.79 (0.73–0.85)	0.612	0.541
OB positive	36 (10.53)	0.68 (0.58–0.78)	0.71 (0.61–0.80)	0.513	0.608
Other minor bleeding	32 (9.36)	0.43 (0.34–0.53)	0.34 (0.26–0.41)	1.799	0.072
All bleeding events	131 (38.30)	0.72 (0.66–0.78)	0.71 (0.65–0.77)	0.467	0.641
Patients with OAC (*n* = 172)					
Major bleeding	4 (2.33)	0.77 (0.61–0.92)	0.83 (0.73–0.94)	0.666	0.506
CRNM GIB	22 (12.79)	0.75 (0.65–0.85)	0.69 (0.57–0.82)	0.825	0.410
OB positive	18 (10.47)	0.66 (0.50–0.81)	0.70 (0.55–0.85)	0.455	0.649
Other minor bleeding	21 (12.21)	0.40 (0.30–0.50)	0.48 (0.36–0.59)	1.075	0.283
All bleeding events	65 (37.79)	0.66 (0.58–0.75)	0.69 (0.61–0.78)	0.597	0.551
Patients with non-OAC (*n* = 170)					
Major bleeding	2 (1.18)	0.60 (0.37–0.83)	0.55 (0.38–0.72)	0.207	0.837
CRNM GIB	35 (20.59)	0.81 (0.73–0.89)	0.80 (0.73–0.88)	0.219	0.827
OB positive	18 (10.59)	0.75 (0.65–0.86)	0.67 (0.55–0.79)	1.568	0.117
Other minor bleeding	11 (6.47)	0.25 (0.12–0.38)	0.37 (0.22–0.53)	1.302	0.193
All bleeding events	66 (38.82)	0.75 (0.67–0.82)	0.76 (0.68–0.83)	0.208	0.836

Note: NVAF, nonvalvular atrial fibrillation; MB, major bleeding; CRNM GIB, clinically relevant nonmajor gastrointestinal bleeding; OB positive, fecal occult blood positive; NAT, no antithrombotic treatment; AP, antiplatelet; VKA, vitamin K antagonists; NOACs, non-vitamin K antagonist; ^#^C-index (95% CI); with OAC, VKA + NOACs; and *Z* statistic from DeLong and others, 1988.

## Data Availability

The data used to support the findings of this study are available from the corresponding author upon request.
